# Human serum enhances the proliferative capacity and immunomodulatory property of MSCs derived from human placenta and umbilical cord

**DOI:** 10.1186/s13287-019-1175-3

**Published:** 2019-03-07

**Authors:** Sermporn Thaweesapphithak, Chairat Tantrawatpan, Pakpoom Kheolamai, Duangrat Tantikanlayaporn, Sittiruk Roytrakul, Sirikul Manochantr

**Affiliations:** 1 Division of Cell Biology, Department of Preclinical Sciences, Faculty of Medicine, Thammasat University, Pathumthani, 12120 Thailand; 2 Center of Excellence in Stem Cell Research, Thammasat University, Pathumthani, 12120 Thailand; 3 Genome Institute, National Center for Genetic Engineering and Biotechnology, National Science and Technology Development Agency, Pathumthani, Thailand

**Keywords:** Mesenchymal stromal cell, Immunosuppression, Human serum, Placenta, Umbilical cord, Con-A, WGA

## Abstract

**Background:**

Mesenchymal stromal cells (MSCs) are considered potential candidates that hold great promise in the treatment of immune-related diseases. For therapeutic applications, it is necessary to isolate and expand MSCs with procedures complying with good manufacturing practice (GMP). Recent studies reported the use of human serum (HS) instead of fetal bovine serum (FBS) for the expansion of bone marrow-derived MSCs. Nevertheless, there are only limited data on HS as an alternative to FBS for the isolation and expansion of umbilical (UC-MSCs) and placenta-derived MSCs (PL-MSCs). In this study, we evaluate the effect of HS compared to FBS on the proliferative and immunosuppressive capacities of these MSCs.

**Methods:**

PL-MSCs and UC-MSCs were isolated and cultured in HS- or FBS-supplemented media. The MSC characteristics, including morphology, immunophenotype, and differentiation ability, were verified. The proliferative and immunosuppressive capacities were also examined. In addition, the proliferative-enhancing factors in both sera were explored using proteomic analysis.

**Results:**

PL-MSCs and UC-MSCs proliferated faster in HS-supplemented medium than in equivalent levels of FBS-supplemented medium. Adipogenic and osteogenic differentiations occurred at nearly identical levels in HS- and FBS-supplemented media. Interestingly, MSCs cultured in HS-supplemented medium had a similar immunosuppressive effect as MSCs cultured in FBS-supplemented medium. Proteomic analysis revealed that Con-A binding glycoproteins with a molecular weight > 100 kDa in FBS could significantly enhance MSC proliferation. In contrast, the proliferative enhancing factors in HS were found in the Con-A non-binding fraction and WGA binding fraction with a molecular weight > 100 kDa.

**Conclusions:**

Taken together, our results suggest applications for the use of HS instead of FBS for the isolation and expansion of PL-MSCs and UC-MSCs for cell therapy in the future. Furthermore, this study identifies factors in HS that are responsible for its proliferative and immunosuppressive effects and might thus lead to the establishment of GMPs for the therapeutic use of MSCs.

## Background

Mesenchymal stromal cells (MSCs), also known as mesenchymal stem cells, are multipotent cells [1] that are commonly characterized by their spindle shape and their ability to adhere on plastic culture plates [2]. As multipotent stem cells, MSCs have the capacity of self-renewal and can differentiate into various mesodermal cell types, including adipocytes, chondrocytes, and osteoblasts [3]. MSCs are widely studied as potential cell therapy agents because of their immunomodulatory effects, which have been established in in vitro studies and in several clinical trials [4, 5]. MSCs thus appear to hold substantial promise for cell therapy, particularly in the treatment of conditions involving autoimmune and inflammatory processes [6–8]. The immunomodulatory properties of MSCs derived from bone marrow (BM-MSCs) have been recognized for a decade [4, 9, 10]. BM-MSCs can suppress T cell proliferation and dendritic cell differentiation, as well as modulate B cell function [7, 11, 12]. Clinical trials of MSC therapy indicated that MSCs can improve the outcome of skin, heart, and kidney transplants [13–16]. MSCs are rare in the BM, especially in elderly donors; therefore, ex vivo expansion is required before they can be used in clinical trials. Apart from BM-MSCs, MSCs derived from placenta (PL-MSCs) and umbilical cord (UC-MSCs) exhibit a similar immunomodulatory and proliferative properties as BM-MSCs. PL-MSCs and UC-MSCs express low alloimmunogenicity, which allows their use as a human leucocyte antigen (HLA)-unmatched off-the-shelf product [17]. This characteristic also makes these cells an ideal candidate for a clinical approach in immune-related diseases. Currently, there is no standard protocol for ex vivo MSC expansion, most of which use fetal bovine serum (FBS) as a supplement. The safety of the materials used in humans is crucial, and a recent study reported that anti-FBS antibodies have been detected in most patients infused with MSCs cultured in the presence of FBS [18]. Moreover, there is an increasing concern regarding transmission of infectious agents from animals to humans, Also, ethical issues related to harvest of the serum, the lot to lot variability of the serum, and an expected shortage of FBS due to routine use in cell therapy have to be considered. Therefore, the use of MSCs in cell therapy requires the development of a GMP (good manufacturing practice) protocol for MSC isolation and expansion. Tremendous efforts have been made by several research groups to establish xeno-free condition for MSC culture [19, 20]. However, the effectiveness of those xeno-free condition has been inconsistent [21, 22] and cannot entirely replace the standard culture condition containing FBS [23]. Thus, suitable culture conditions for clinical scale manufacturing of MSCs still remain a crucial matter. Recently, human serum (HS) has been suggested as an alternative to FBS [18]. Human serum contains abundant bioactive compounds and growth factors such as platelet-derived growth factor (PDGF) AA/AB that can enhance MSC proliferation without altering MSC characteristics and functional properties [24]. Recent studies have addressed the effect of HS on the expansion of BM-MSCs and adipose tissue-derived MSCs. MSCs expanded in HS-containing media had a similar phenotype and functional properties as MSCs cultured in FBS-containing media [18, 25]. There are limited data available on the effect of HS on the proliferative and immunosuppressive properties of PL-MSCs and UC-MSCs. These data are however required in view of an alternative source of MSCs expanded in an animal-free system for the potent immunosuppressive effect exerted by alloreactive T cells in the hematopoietic stem cell transplantation (HSCT) setting. The aims of the study were first to compare the effect of HS- and FBS-supplemented media on the biological characteristics and immunosuppressive property of PL-MSCs and UC-MSCs. Secondly, we explored the proliferation enhancing factors in HS in comparison to FBS in order to establish xeno-free factors for therapeutic uses.

## Materials and methods

### Collection of human samples

This study was approved by the Human Research Ethics Committee of Thammasat University No.I (Faculty of Medicine) and is in accordance with the declaration of Helsinki and Belmont report. All samples were obtained from donors with written informed consent. The placentas and umbilical cords were taken from pregnant women after delivery at Thammasat Chalermprakiat Hospital. Peripheral blood was obtained from healthy volunteers. Subjects that had any clinical history of malignancy, metabolic disorder, or infectious disease were excluded from the study.

### Preparation of human serum

From each donor, 20 ml of blood was taken without anticoagulant and allowed to clot overnight at 4 °C. After centrifugation at 2000×*g* for 30 min, the serum was filtered through 0.22-μm filters (Millipore, USA). The pooled serum was aliquoted and frozen at − 20 °C. After thawing, the serum was centrifuged to remove the aggregated material and then maintained at 4 °C until use.

### Isolation and expansion of MSCs

The placentas and umbilical cords (*n* = 5) were taken from pregnant women after delivery at Thammasat Chalermprakiat Hospital. Placental tissue (size ~ 3 × 3 × 3 cm) or umbilical cord (length ~ 2–4 cm) were chopped into small pieces and digested with 1.6 mg/ml collagenase IV (Sigma-Aldrich, USA) and 200 mg/ml deoxyribonuclease I (Sigma-Aldrich, USA) for 4 h at 37 °C. After washing twice with phosphate-buffered saline (PBS), the cells were cultured in MSC growth medium: Dulbecco’s modified Eagle medium (DMEM; GibcoBRL, USA) supplemented with either 10% HS or 10% FBS (GibcoBRL, USA). The cultures were maintained at 37 °C in a humidified tissue culture incubator containing 5% CO_2_. The medium was replaced twice a week. For further expansion, the plastic-adherent cells were sub-cultured using 0.25% trypsin-EDTA (Invitrogen, USA) and re-plated at density of 1 × 10^4^cells/cm^2^. Cells from passage 3 to 5 were used for all experiments.

### Immunophenotype of MSCs

MSCs cultured in DMEM supplemented with either FBS or HS were trypsinized using 0.25% trypsin-EDTA. The cell suspensions were stained with phycoerythrin (PE)- or fluorescein isothiocyanate (FITC)-conjugated antibodies against-human CD34 (Bio Legend, USA), CD45 (Bio Legend, USA), CD73 (Bio Legend, USA), CD90 (Bio Legend, USA), or CD105 (BD Bioscience, USA) for 30 min at 4 °C. Subsequently, the cells were fixed with 1% paraformaldehyde in PBS. For each marker, 20,000 events were acquired and analyzed using flow cytometry (FACScalibur™, Becton Dickinson, USA) and CellQuest® software (Becton Dickinson, USA).

### Differentiation potential of MSCs

For adipogenic differentiation, 7.5 × 10^4^ MSCs cultured in DMEM supplemented with either FBS or HS were seeded into 35-mm^2^ dishes (Costa, Corning, USA) containing MSC growth medium and allowed to adhere to the plate overnight. Subsequently, growth medium was replaced with adipogenic differentiation medium: DMEM supplemented with 10% FBS, 500 μM isobutylmethylxanthine (Sigma-Aldrich, USA), 200 μM indomethacin (Sigma-Aldrich, USA), 25 mM glucose, 1 μM dexamethasone, and 10 μM insulin (Sigma-Aldrich, USA). The medium was replaced twice a week. After 4 weeks, the cells were washed with PBS and fixed with 4% formaldehyde. The cells were then stained with 0.3% Oil Red O (Sigma-Aldrich, USA) in 60% isopropanol for 20 min and observed using an inverted microscope (Nikon TS100, Japan).

For osteogenic differentiation, 4.5 × 10^4^ MSCs were seeded into 35-mm^2^ dishes containing MSC growth medium and left overnight. Then, the medium was removed and substituted by osteogenic differentiation medium: DMEM supplemented with 10% FBS, 0.1 μM dexamethasone, and 300 μM ascorbic acid. The medium was replaced every 3 days. On culture day 7 onward, 10 mM β-glycerophosphate was added into the osteogenic differentiation medium. After culture for 4 weeks, the cells were washed twice with PBS, fixed with 4% paraformaldehyde, and stained with Alizarin Red S (Sigma-Aldrich, USA) for 30 min.

For control, cells were maintained in MSC growth medium and processed similar to the cells in the adipogenic or osteogenic differentiation media, respectively.

### Growth kinetics of MSCs

To determine the effect of HS compared to FBS on MSC expansion, 1 × 10^3^ culture-expanded MSCs (passage 2–4) were seeded into an individual well of 24-well plates (Costa, corning, USA) containing MSC growth medium supplemented with either 10% HS or 10% FBS. The cultures were maintained at 37 °C in a humidified tissue culture incubator with 5% CO_2_. The cell number was determined using hematocytometer. The mean numbers of cells were calculated and plotted against culture time to generate a growth curve. The population doubling time assay was also performed for each isolated cell population. The means of the triplicate cell counts for each passage were calculated and plotted against culture time to generate a population doubling time curve.

### Immunosuppressive effect of MSCs

To examine the inhibitory effect of MSCs expanded with HS on T cell proliferation, 2 × 10^4^ MSCs were seeded in triplicate into an individual well of 96-well plates containing 100 μl of MSC growth medium supplemented with either 10% HS or FBS. On the following day, 2 × 10^4^ peripheral blood mononuclear cells (PB-MNCs) from the interphase layer of heparinized blood were stimulated with 2% phytohaemagglutinin (PHA, Thermo Scientific, USA) and added to the plates containing MSC cultures in RPMI 1640 medium (Thermo Scientific, USA) supplemented with either 10% HS or FBS. Co-culture of MSCs and PB-MNCs without PHA was used as control. After 5 days of co-culture, 100 μl of cell suspension from each well was collected and incubated with 10 μl of Cell Counting Kit-8 (Dojindo, Japan) for 4 h at 37 °C. The absorbance at 450 nm was measured using a microplate reader (Biotek Powerwave XS; BioTex, USA) to determine cell number. The proliferative index was calculated by the following equation:

$$ \mathrm{Proliferative}\ \mathrm{index}=\frac{\left(\mathrm{O}.\mathrm{D}.\mathrm{sample}-\mathrm{O}.\mathrm{D}.\mathrm{blank}\right)}{\left(\mathrm{O}.\mathrm{D}.\mathrm{control}-\mathrm{O}.\mathrm{D}.\mathrm{blank}\right)} $$

### Expression of *IDO*, *COX-2*, and *iNOS*

To explore the mechanism that MSCs cultured in HS use to inhibit activated T cell proliferation, 2 × 10^5^ MSCs were seeded into an individual well of six-well plates (Costa, Corning, USA) containing MSCs growth medium supplemented with either 10% HS or FBS. On the following day, the medium was removed and 2 × 10^5^ PHA-activated PB-MNCs or fresh medium containing 10 ng/ml interferon-γ (IFN-γ; Peprotech, USA) were added. Cultures of MSCs alone was used as controls and carried out in parallel to the experiments.

After 96 h of incubation, total RNA was extracted from the cultured MSCs using the RNeasy Mini Kit (QIAGEN, Germany) and cDNA was generated using the SuperScript® III First Strand Synthesis Kit (Invitro-gen, USA). The expression levels of indoleamine 2,3-dioxygenase (*IDO*), cyclooxygenase-2 (*COX-2*), and inducible nitric oxide synthase (*iNOS*) were determined by quantitative real-time polymerase chain reaction (qRT-PCR) using a Step one plus™ Real-Time PCR system (Applied Biosystems; ABI, USA). Primer sequences are shown in Table 1. The quantitation of each target gene was normalized with the quantitation glyceraldehyde-3-phosphate dehydrogenase (*GAPDH*). The data were analyzed by comparative ^ΔΔ^CT method using StepOne™ Software version 2.2 and presented as the relative mRNA expression level. Each sample was examined in triplicate and the mean value was calculated.

**Table 1:** Primer sequences and the amplicon sizes

Gene	Forward primer	Reverse primer	Amplicon size
*IDO*	5′-GGCAAAGGTCATGGAGATGT-3′	5′-TCCAGTTTGCCAAGACACAG-3′	127
*COX-2*	5′-GACTCCCTTGGGTGTCAAAG-3′	5′-AACTGATGCGTGAAGTGCTG-3′	147
*iNOS*	5′-CTCTATGTTTGCGGGGATGT-3′	5′-TTCTTCGCCTCGTAAGGAAA-3′	179
*GAPDH*	5′-GTCAACGGATTTGGTCGTATTG-3′	5′-CATGGGTGGAATCATATTGGAA-3′	193

### Western blot analysis

MSCs derived from the placenta and umbilical cord (1 × 10^6^ cells) were cultured in 25-cm^2^ tissue cultured flasks containing MSC growth medium supplemented with either 10% HS or FBS. On the following day, the medium was removed and 1 × 10^6^ PHA-activated PB-MNCs or fresh medium containing 10 ng/ml of IFN-γ were added. Cultures of MSCs alone was used as control and carried out in parallel to the experiments. After 72 h, the cultured MSCs were trypsinized and lyzed in RIPA buffer (Amresco®, USA) containing 1 mM phenylmethane sulfonyl fluoride (PMSF, Sigma-Aldrich, USA) and 1X protease inhibitor cocktail (Amresco®, USA) for 10 min at 4 °C. After centrifugation, the supernatant was collected and protein concentration was determined using Bio-Rad Protein Assay (Bio-Rad, USA).

Proteins were then separated on a 12% SDS polyacrylamide gel and transferred onto nitrocellulose membrane (Hybond ECL; Amersham Pharmacia, USA) using Trans-Blot® SD Semi-Dry Transfer Cell (Bio-Rad, USA).

Following transfer, the membrane was incubated in the blocking solution, 10% skim milk in Tris-buffered saline containing 0.1% Tween 20 (TBST) for 1 h with agitation at room temperature. Primary antibody against IDO (Sigma-Aldrich, USA) was diluted in TBST containing 3% bovine serum albumin (BSA) at a dilution of 1:250. The membrane was then incubated overnight at 4 °C followed by washing with TBST three times, 10 min each. The membrane was then incubated with an HRP-conjugated goat anti-mouse IgG (Sigma-Aldrich, USA) at a dilution of 1:2000 in TBST-BSA for 45 min at room temperature, washed with TBST three times, 10 min each. The signal was visualized using SuperSignal™ West Pico Chemiluminescent Substrate (Thermo Scientific, USA) and detected by Odyssey Fc Imaging System (Li-COR, USA). After normalizing with actin, the densitometric value from three independent experiments was expressed as the mean ± SEM.

### Cytokine inhibition assays

MSCs derived from placenta and umbilical cord (2 × 10^4^ cells) were plated as triplicate into 96-well plates containing 100 μl of MSC growth medium supplemented with either 10% HS or FBS and allowed to adhere to the plates overnight. Thereafter, 100 μl of PHA-activated PB-MNCs (1 × 10^5^ cells/ml) were added into each MSC-containing wells. To study the role of IDO, COX-2 and iNOS in the immunosuppressive effect of MSCs cultured in HS, 500 μM 1-methyl-l-tryptophan (1-MT; Sigma-Aldrich, USA), 20 μM indomethacin (Sigma-Aldrich, USA), and 1 mM *N*-nitro-l-arginine methyl ester (L-NAME, Sigma-Aldrich, USA) were added to suppress the activities of IDO, COX-2 and iNOS, respectively, as previously described [26]. After 5 days of culture, 100 μl of cell suspension from each well was transferred to new 96-well plates and 10 μl of Cell Counting Kit-8 was added. After incubating at 37 °C for 4 h, the absorbance at 450 nm was measured and the proliferative index was calculated.

### Serum fractionation

To explore the essential factors in the serum, HS and FBS were fractionated using Macrosep® Advance Centrifugal Devices (Pall Corporation, USA) with a molecular weight cut-off of 100 kDa, 30 kDa, 10 kDa, and 3 kDa. Briefly, HS or FBS was added into sample reservoir (100 kDa) and centrifuged at 10,000×*g* for 10 min. The sample retained in sample reservoir (fraction > 100 kDa) was transferred to a new centrifuge tube (Costa, Corning, USA), and the sample in filtrate receiver was transferred to next centrifugal devices, 30 kDa, 10 kDa, and 3 kDa, respectively. The fractions in sample reservoirs were collected, 30–100 kDa, 10–30 kDa, 3–10 kDa, and < 3 kDa. The protein concentration of each fraction was measured using the Bradford assay and kept at − 80 °C until use.

### The effect of fractionated serum on MSC proliferation

To study the effect of fractionated HS/FBS on MSC proliferation, MSCs derived from placenta and umbilical cord were seeded at a density of 500 cells/cm^3^ in 24-well plate containing 500 μl of DMEM supplemented with either 5% FBS or HS. Proteins from each fractions (< 3 kDa, 3–10 kDa, 10–30 kDa, 30–100 kDa, and > 100 kDa) were added into the cultures at a concentration of 35 μg/ml. MSCs cultured in DMEM supplemented with either 10% FBS or HS were served as a control. The cultures were maintained at 37 °C in a humidified tissue culture incubator with 5% CO_2_ for 10 days. The number of cells in culture was counted at several intervals (0, 3, 5, 7, and 10 days) using hematocytometer. The mean number of cells was calculated and plotted against culture time to generate a growth curve.

### Enrichment of serum glycoprotein using affinity column chromatography

To investigate the factors involved in MSC proliferation, the serum fraction containing protein whose molecular weight > 100 kDa was further fractionated with a glycoprotein isolation kit using either Concanavalin A (Con-A; Thermo Scientific, USA) or Wheat Germ Agglutinin (WGA; Thermo Scientific, USA) according to the manufacturer’s instructions.

Briefly, 5X binding/wash buffer stock solution was added to the > 100 kDa fraction at a ratio of 1:4. After mixing, the sample was added to either a Con-A or a WGA lectin resin column and incubated for 10 min at room temperature with end-over-end mixing using a rotator. Thereafter, the columns were centrifuged at 1000×*g* for 1 min, and the flow-through fraction was collected as Con-A or WGA non-binding fractions. Then, the columns were washed with 1X binding/wash buffer two times. Subsequently, the 200 μl elution buffer was added and incubated for 5 min at room temperature. After centrifugation at 1000×*g* for 1 min, the eluted fraction was collected as Con-A or WGA binding fractions. All serum sub-fractions were then desalted using ÄKTA™ start Grundgerät (VWR International GmbH, Germany) and Bio-Scale™ Mini Bio-Gel® P-6 Desalting Cartridges (Bio-Rad, USA). The protein concentration was measured using the Bradford assay. These fractions, Con-A binding fraction, Con-A non-binding fraction, WGA binding fraction, and WGA non-binding fraction were tested for effects on MSCs proliferation by the methods mentioned above.

### Statistical analysis

All experiments were performed in triplicate. The data were presented as mean ± standard error of mean (SEM). Statistical comparison was performed using the paired *T* test for paired samples. A *p*-value of less than 0.05 was considered to be statistically significant.

## Results

### Morphology of MSCs

After initial seeding for 3 days, placenta-derived MSCs (PL-MSCs) cultured in HS-supplemented medium could attach and spread on the plastic surface of the tissue culture flasks. The adherent cells exhibited an elongated, spindle-shaped morphology similar to that of the cells cultured in FBS-supplemented medium. After sub-culturing, the cells maintained in HS-supplemented medium proliferated rapidly and reached 80% confluence within 2 weeks, similar to the cells maintained in FBS-supplemented medium (Fig. 1a). PL-MSCs could be expanded in HS-supplemented medium for more than 20 passages without any noticeable changes in their morphology, similar to that of PL-MSCs expanded in FBS-supplemented medium.

**Fig. 1:** The characteristics of MSCs derived from human placenta (PL-MSCs) and umbilical cord (UC-MSCs) cultured in human serum (HS) compared to fetal bovine serum (FBS). **a** The spindle-shaped morphology of PL-MSCs and UC-MSCs. **b** Flow cytometry demonstrated the expression of typical MSC markers. The percentage of positive cells was not significantly different from each other whether they were cultured in HS- or FBS-supplemented medium. Data are presented as mean ± SEM. **c** The adipogenic and osteogenic differentiation potentials of PL-MSCs and UC-MSCs

For umbilical cord-derived MSCs (UC-MSCs), the cells cultured in HS-supplemented medium also exhibited an elongated, spindle-shaped morphology similar to that of the cells cultured in FBS-supplemented medium. After passaging, the cells maintained in HS-supplemented medium proliferated rapidly and reached 80% confluence within 2 weeks similar to the cells maintained in FBS-supplemented medium (Fig. 1a). UC-MSCs could be expanded in HS-supplemented medium for more than 20 passages without any apparent changes in their morphology, similar to that of UC-MSCs expanded in FBS-supplemented medium.

### Immunophenotype of MSCs

The expression of typical MSC markers in PL-MSCs and UC-MSCs cultured in HS-supplemented medium were examined and compared to that of MSCs cultured in FBS-supplemented medium. The results demonstrated that PL-MSCs and UC-MSCs cultured in HS-supplemented medium expressed typical MSC markers including CD73, CD90, and CD105. They did not express hematopoietic markers such as CD34 and CD45 similar to PL-MSCs and UC-MSCs cultured in FBS-supplemented medium (Fig. 1b). The percentages of cells which expressed these markers were not significantly different whether the cells were cultured in either HS- or FBS-supplemented medium (Fig. 1b).

### Adipogenic differentiation potential of MSCs

To examine the adipogenic differentiation potential of MSCs cultured in HS-supplemented medium compared to MSCs cultured in FBS-supplemented medium, PL-MSCs and UC-MSCs cultured in either HS- or FBS-supplemented medium were harvested and cultured in adipogenic differentiation medium. After culture for 4 weeks, cell morphology transformed from spindle-shaped cells to bulky round cells. Numerous lipid droplets positive for Oil Red O were observed in the cytoplasm of both PL-MSCs and UC-MSCs cultured in HS-supplemented medium, similar to those of the cells cultured in FBS-supplemented medium (Fig. 1c). Control PL-MSCs and UC-MSCs cultured in either HS- or FBS-supplemented medium throughout the entire cultured period maintained their fibroblast-like morphology without generating any lipid droplets, and they were negative for Oil Red O staining.

### Osteogenic differentiation potential of MSCs

To study the osteogenic differentiation potential of MSCs cultured in HS-supplemented medium compared to MSCs cultured in FBS-supplemented medium, PL-MSCs and UC-MSCs cultured in either HS- or FBS-supplemented medium were harvested and cultured in osteogenic differentiation medium. After 4 weeks, PL-MSCs and UC-MSCs cultured in HS-supplemented medium differentiated into osteoblast-like cells similar to those of the cells cultured in FBS-supplemented medium. Alizarin Red S stained extracellular calcium deposits in these cell cultures, proving their osteogenic activity (Fig. 1c). On the other hand, PL-MSCs and UC-MSCs cultured in either HS- or FBS-supplemented medium throughout the entire cultured period maintained their fibroblast-like morphology without generating any osteoblast-like cells and they produced no calcium deposits that could be stained by Alizarin Red S.

### Growth kinetics of MSCs cultured in human serum

To examine the growth kinetics of MSCs cultured in HS-supplemented medium compared to MSCs cultured in FBS-supplemented medium, PL-MSCs and UC-MSCs at the second to fourth passage were seeded into 24-well plates containing MSC growth medium supplemented with either 10% FBS or HS. The cells were harvested at days 1 to 7 to determine the cell number. The result showed that at the second passage, the cell numbers of both PL-MSCs and UC-MSCs cultured in either HS- and FBS-supplemented medium was not different. At the third and fourth passages, the cell number of PL-MSCs cultured in HS-supplemented medium was significant higher than that of PL-MSCs cultured in FBS-supplemented medium (*p* < 0.05, Fig. 2). PL-MSCs cultured in HS-supplemented medium could expand about 40-fold within 7 days whereas PL-MSCs cultured in FBS-supplemented medium could expand only about 20-fold within 7 days. Similar to PL-MSCs, at the third and fourth passages, the cell number of UC-MSCs cultured in HS-supplemented medium was significantly higher than that of UC-MSCs cultured in FBS-supplemented medium (*p* < 0.05, Fig. 2). UC-MSCs cultured in HS-supplemented medium could expand about 60-fold within 7 days whereas UC-MSCs cultured in FBS-supplemented medium could expand only about 42-fold within 7 days.

**Fig. 2:** Growth kinetics of PL-MSCs (**a**, **c**, **e**, **g**) and UC-MSCs (**b**, **d**, **f**, **h**) cultured in MSC growth medium supplemented with 10% HS compared to PL-MSCs and UC-MSCs cultured in MSC growth medium supplemented with 10% FBS. Data from three independent experiments were presented as mean ± standard error of the means (SEM). *p < 0.05 compared with MSCs cultured in FBS

Furthermore, population doubling times of the cells were determined in the cells harvested at culture day 7. The results showed that the population doubling times of PL-MSCs and UC-MSCs cultured in either HS- or FBS-supplemented medium at the second passage were not different. At the third and fourth passages, the population doubling time of PL-MSCs cultured in HS-supplemented medium was significantly shorter than that of PL-MSCs cultured in FBS-supplemented medium. Similar to PL-MSCs, at the third and fourth passages, the population doubling time of UC-MSCs cultured in HS-supplemented medium was significantly shorter than that of UC-MSCs cultured in FBS-supplemented medium (Fig. 2).

### The immunosuppressive effect of MSCs on T cell proliferation

#### The effect of MSCs on activated T cell proliferation

The proliferative index of PHA-activated T cells co-cultured with PL-MSCs-HS was significantly decreased when compared to PHA-activated T cells alone (Fig. 3a). For UC-MSCs, the proliferative index of PHA-activated T cells co-cultured with UC-MSCs-HS was also significantly decreased when compared to the culture of PHA-activated T cells alone (Fig. 3b). Interestingly, the proliferative index of PHA-activated T cells co-cultured with either PL-MSCs-HS or UC-MSCs-HS was not difference from that of PHA-activated T cells co-cultured with either PL-MSCs-FBS or UC-MSCs-FBS, respectively. Therefore, MSCs cultured in human serum can inhibit the proliferation of activated T cells to the same degree as MSCs cultured in fetal bovine serum.

**Fig. 3:** The immunosuppressive effect of PL-MSCs (**a**) and UC-MSCs (**b**) on PHA-activated T cell proliferation. *p < 0.05 compared to PHA-activated T cells. *p < 0.05: significant difference compared to MNCs-PHA

#### The expression of genes involved in the immunosuppressive capacity of MSCs

Quantitative real-time PCR (qRT-PCR) was performed to examine the expression level of genes involved in immunosuppression including indoleamine 2, 3-dioxygenase (*IDO*), cyclooxygenase-2 (*COX-2*), and inducible nitric oxide synthase (*iNOS*). The results are the following:

##### Expression of indoleamine 2,3-dioxygenase

The expression of *IDO* was significantly increased in PL-MSCs-FBS co-cultured with PHA-activated T cells compared to that in PL-MSCs-FBS without PHA-activated T cells (Fig. 4a). Similar to PL-MSCs-FBS, PL-MSCS-HS co-cultured with PHA-activated T cells had a significantly higher *IDO* expression than PL-MSCs-HS cultured without PHA-activated T cells (Fig. 4a). In addition, the expression of *IDO* was significantly increased in UC-MSCs-FBS co-cultured with PHA-activated T cells compared to UC-MSCs-FBS without PHA-activated T cells (Fig. 4a). UC-MSCs-HS co-cultured with PHA-activated T cells had significantly higher *IDO* expression than UC-MSCs-HS cultured without PHA-activated T (Fig. 4a).

**Fig. 4:** **a**–**c** Mean value of relative gene expression in MSCs co-cultured with PHA-activated T cells or IFN-γ. Data are presented as mean ± standard error of the means. *p < 0.05: significant difference compared to MSCs. ^#^*p* < 0.05: significant difference compared to MSCs+MNCs+PHA. ^+^*p* < 0.05: significant difference compared to MSCs-FBS+IFN-γ

To determine the factors secreted by activated T cells that could induce the expression of *IDO*, experiments were performed by adding the pro-inflammatory cytokine, IFN-γ, to the culture of MSCs. IFN-γ can significantly enhance the expression of *IDO* in PL-MSCs-FBS and PL-MSCs-HS compared to PL-MSCs-FBS and PL-MSCs-HS cultured without IFN-γ (Fig. 4a). Interestingly, PL-MSCs-FBS and PL-MSCs-HS cultured with IFN-γ had significantly higher *IDO* expression than PL-MSCs-FBS and PL-MSCs-HS co-cultured with PHA-activated T cells. Similar to PL-MSCs, UC-MSCs-FBS and UC-MSCS-HS cultured with IFN-γ had significantly higher *IDO* expression than UC-MSCs-FBS and UC-MSCs-HS cultured without IFN-γ (Fig. 4a). Remarkably, UC-MSCs-FBS and UC-MSCs-HS cultured with IFN-γ had significantly higher *IDO* expression than UC-MSCs-FBS and UC-MSCs-HS co-cultured with PHA-activated T cells (Fig. 4a). It should be noted that the expression of *IDO* in MSCs cultured with HS-supplemented medium was not significantly different than that of MSCs cultured with FBS-supplemented both in IFN-γ stimulated MSCs and activated T cells stimulated MSCs.

##### Expression of cyclooxygenase-2

The stimulation of PL-MSCs-FBS with PHA-activated T cells significantly increased the expression of *COX-2* in comparison with PL-MSCs-FBS cultured without PHA-activated T cells (Fig. 4b). Similar to PL-MSCs-FBS, PL-MSCS-HS co-cultured with PHA-activated T cells had significantly higher *COX-2* expression than PL-MSCs-HS cultured without PHA-activated T cells (Fig. 4b). In addition, the expression of *COX-2* was significantly increased in UC-MSCs-FBS co-cultured with PHA-activated T cells (Fig. 4b). UC-MSCs-HS co-cultured with PHA-activated T cells had significantly higher *COX-2* expression than UC-MSCs-HS cultured without PHA-activated T cells (Fig. 4b). IFN-γ could not enhance the expression of *COX-2* in both PL-MSCs-FBS and PL-MSCs-HS when compared to PL-MSCs-FBS and PL-MSCs-HS cultured without IFN-γ (Fig. 4b). Similar to PL-MSCs, UC-MSCs-FBS and UC-MSCs-HS cultured with IFN-γ showed no significant difference in *COX-2* expression when compared to UC-MSCs-FBS and UC-MSCs-HS cultured without IFN-γ (Fig. 4b). Interestingly, PL-MSCs-FBS and PL-MSCs-HS cultured with IFN-γ had significantly lower *COX-2* expression than PL-MSCs-FBS and PL-MSCs-HS co-cultured with PHA-activated T cells. Similar to PL-MSCs, UC-MSCs-FBS and UC-MSCs-HS cultured with IFN-γ had significantly lower *COX-2* expression than UC-MSCs-FBS and UC-MSCs-HS co-cultured with PHA-activated T cells (Fig. 4b). It should be noted that the expression of *COX-2* in MSCs cultured with HS-supplemented medium was not significantly different compared to MSCs cultured with FBS-supplemented medium both in IFN-γ stimulated MSCs and activated T cells stimulated MSCs.

##### Expression of inducible nitric oxide synthase

The expression of *iNOS* was significantly increased in PL-MSCs-FBS co-cultured with PHA-activated T cells compared to PL-MSCs-FBS without PHA-activated T cells (Fig. 4c). In contrast to PL-MSCs-FBS, the expression of *iNOS* in PL-MSCs-HS co-cultured with PHA-activated T cells was not different from PL-MSCs-HS cultured without PHA-activated T cells (Fig. 4c). In UC-MSCs, the expression of *iNOS* was significantly increased in UC-MSCs-FBS co-cultured with PHA-activated T cells compared to UC-MSCs-FBS without PHA-activated T cells (Fig. 4c). Interestingly, both PL-MSCs-HS and UC-MSCs-HS co-cultured with PHA-activated T cells had significantly lower *iNOS* expression compared to PL-MSCs-FBS and UC-MSCs-FBS co-cultured with PHA-activated T cells, respectively.

Furthermore, IFN-γ significantly enhanced the expression of *iNOS* in PL-MSCs-FBS and PL-MSCs-HS when compared to PL-MSCs-FBS and PL-MSCs-HS cultured without IFN-γ, respectively (Fig. 4c). Similar to PL-MSCs, UC-MSCs-FBS and UC-MSCS-HS cultured with IFN-γ had significantly higher *iNOS* expression than UC-MSCs-FBS and UC-MSCs-HS cultured without IFN-γ (Fig. 4c). Interestingly, PL-MSCs-HS and UC-MSCs-HS cultured with IFN-γ had significantly higher *iNOS* expression than PL-MSCs-FBS and UC-MSCs-FBS cultured with IFN-γ. Remarkably, PL-MSCs-FBS and UC-MSCs-FBS co-cultured with PHA-activated T cells had significantly higher *iNOS* expression than the cells cultured with IFN-γ (Fig. 4c). In contrast, PL-MSCs-HS and UC-MSCs-HS cultured with IFN-γ had significantly higher *iNOS* expression than the cells co-cultured with PHA-activated T cells (Fig. 4c).

#### Protein expression involved in the immunosuppressive capacity of MSCs

The results of gene expression indicated that *IDO* has the highest expression level; therefore, the expression of IDO at the protein levels was confirmed using Western blot analysis (Fig. 5a). The result of protein expression was coincident with the gene expression. The level of IDO protein expression was significantly increased in PL-MSCs-FBS co-cultured with activated T cells compared to PL-MSCs-FBS cultured without activated T cells (Fig. 5b). In addition, IFN-γ significantly enhanced IDO expression compared to PL-MSCs-FBS cultured without IFN-γ (Fig. 5b). Similar to PL-MSCs-FBS, the level of IDO protein expression was significantly increased in PL-MSCs-HS co-cultured with activated T cells compared to PL-MSCs-HS cultured without activated T cells (Fig. 5b). In addition, IFN-γ significantly enhanced IDO expression in PL-MSCs-FBS compared to PL-MSCs-HS cultured without IFN-γ (Fig. 5b). Interestingly, PL-MSCs cultured in HS had significantly higher IDO expression than PL-MSCs cultured in FBS (Fig. 5b).

**Fig. 5:** **a**, **b** The expression level of IDO protein in PL-MSCs and UC-MSCs co-cultured with PHA-activated T cells or IFN-γ. *p < 0.05: significant difference compared to MSCs. #*p* < 0.05 compared to MSCs cultured in FBS-supplemented medium

In UC-MSCs, the level of IDO protein expression was significantly increased in UC-MSCs-FBS co-cultured with activated T cells in comparison with UC-MSCs-FBS cultured without activated T cells (Fig. 5b). In addition, IFN-γ significantly enhanced IDO expression in UC-MSCs-FBS compared to UC-MSCs-FBS cultured without IFN-γ. Similar to UC-MSCs-FBS, the level of IDO protein expression was significantly increased in UC-MSCs-HS co-cultured with activated T cells in comparison with UC-MSCs-HS cultured without activated T cells (Fig. 5b). In addition, IFN-γ significantly enhanced IDO expression in UC-MSCs-HS compared to UC-MSCs-HS which were cultured without IFN-γ (Fig. 5b). Interestingly, UC-MSCs cultured in HS had significantly higher IDO expression than UC-MSCs cultured in FBS (Fig. 5b).

##### Immunosuppressive capacity of MSCs after cytokine inhibition

To further confirm the role of the soluble factors, IDO, COX-2, and iNOS, on MSC-mediated immune suppression, the inhibition assay was performed using chemical antagonists to those cytokines, 1-MT for IDO, indomethacin for COX-2, and L-NAME for iNOS. The results demonstrated that the proliferative indices of PHA-activated T cells co-cultured with PL-MSCs-FBS in the presence of 1-MT, indomethacin, or L-NAME were significantly increased when compared to PHA-activated T cells cocultured with PL-MSCs-FBS without chemical antagonists.

However, the proliferative indices of these PHA-activated T cells did not reverse to the level of the positive control (MNCs+PHA). Similar to PL-MSCs-FBS, the proliferative indices of PHA-activated T cells co-cultured with PL-MSCs-HS in the presence of 1-MT, indomethacin, or L-NAME were also significantly increased compared to PHA-activated T cells co-cultured with PL-MSCs-HS without chemical antagonists. Again, the proliferative indices of these PHA-activated T cells did not reverse to the level of the positive control (MNCs+PHA) (Fig. 6a).

**Fig. 6:** The effect of cytokine inhibition on the immunosuppressive effect of PL-MSCs (**a**) and UC-MSCs. (**b**). PHA-activated T cells were co-cultured with either MSCs-FBS or MSCs-HS in the presence or absence of the specific antagonists 1-MT, indomethacin, or L-NAME. Data are presented as mean ± SEM from three independent experiments. *p < 0.05: significant difference compared to MNCs+PHA+MSCs-FBS. ^#^*p* < 0.05: significant difference compared to MNCs+PHA+MSCs-HS

Similar to PL-MSCs, the proliferative index of PHA-activated T cells co-cultured with UC-MSCs-FBS in the presence of 1-MT, indomethacin, or L-NAME was significantly higher than that of PHA-activated T cells co-cultured with UC-MSCs-FBS without chemical antagonists. And again, the proliferative indices of these PHA-activated T cells did not reverse to the level of the positive control (MNCs+PHA) (Fig. 4b). Similar to UC-MSCs-FBS, the proliferative index of PHA-activated T cells co-cultured with UC-MSCs-HS in the presence of 1-MT, indomethacin, or L-NAME was also significantly higher than that of PHA-activated T cells co-cultured with UC-MSCs-HS without chemical antagonists, but again, they did not reverse to the level of the positive control (MNCs+PHA) (Fig. 6b).

Interestingly, adding two or three chemical antagonists to the co-culture of PHA-activated T cells and MSCs showed similar levels of immunosuppression compared to adding only one chemical antagonist (Fig. 6). Taken together, the immunosuppressive effect of PL-MSCs and UC-MSCs cultured in human serum might be mediated, at least in part, through IDO, COX-2, and iNOS similar to that of PL-MSCs and UC-MSCs cultured in fetal bovine serum. However, the fact that an inhibition of IDO, COX-2, and iNOS activities failed to abolish the immunosuppressive effect of PL-MSCs and UC-MSCs suggests that PL-MSCs and UC-MSCs can also mediate immunosuppression through other additional unidentified factors, apart from IDO, COX-2, and iNOS.

### Proteomic analysis of human serum and fetal bovine serum

The growth kinetic results suggested that HS had a positive effect on MSC growth; therefore, the proteome of HS was further characterized to identify the essential factors that enhance MSC growth. In addition, the proteome of FBS was also characterized and compared to that of HS.

#### The effect of fractionated human serum on MSCs growth

To identify the proliferation enhancing factors in HS, the serum was initially fractionated according to the molecular weight into five distinct fractions including < 3 kDa, 3–10 kDa, 10–30 kDa, 30–100 kDa, and > 100 kDa. The effect of each fraction on MSC growth was then investigated using the proliferation assay. Unfractionated HS (10% HS) was used as a positive control while 5% HS was used as a negative control. The results showed that the > 100 kDa fraction of HS induced significantly higher numbers of PL-MSCs compared to unfractionated HS (Fig. 7c). While the fractions of < 3 kDa, 3–10 kDa, 10–30 kDa, and 30–100 kDa of HS could increase PL-MSC growth when compared to the negative control, the proliferation of PL-MSCs induced by these fractions was still lower than that induced by unfractionated HS (Fig. 7c).

**Fig. 7:** The effect of fractionated serum on MSC proliferation. PL-MSCs (**a**, **c**) and UC-MSCs (**b**, **d**) were cultured in DMEM+ 5% serum supplemented with < 3 kDa, 3–10 kDa, 10–30 kDa, 30–100 kDa, or > 100 kDa fractions. The unfractionated serum (10% serum) served as a positive control while 5% serum served as a negative control. Data are presented as mean ± SEM from three independent experiments. *p < 0.05 compared to 10% serum

Similar to PL-MSCs, the > 100 kDa fraction of HS could induce significantly higher numbers of UC-MSCs compared to unfractionated HS (Fig. 7d). Although the fractions of < 3 kDa, 3–10 kDa, 10–30 kDa, and 30–100 kDa in HS could increase UC-MSCs growth when compared to the negative control, the proliferation of UC-MSCs induced by these fractions was still lower than that induced by unfractionated human serum (Fig. 7d).

Taken together, the results suggested that the > 100 kDa fraction of HS induced the highest number of MSCs and thus might contain proliferation enhancing factors; therefore, the > 100 kDa fraction was selected for further analysis.

#### The effect of fractionated fetal bovine serum on MSCs growth

To identify the proliferation enhancing factors in FBS, the serum was initially fractionated according to the molecular weight into five distinct fractions (< 3 kDa, 3–10 kDa, 10–30 kDa, 30–100 kDa, and > 100 kDa) similar to HS. The effect of each fraction on MSC growth was then investigated using the proliferation assay. The unfractionated FBS (10% FBS) served as a positive control while 5% FBS served as a negative control. The results were coincident with those of HS. At the end of culture period, the > 100 kDa fraction of FBS induced significantly higher numbers of PL-MSCs compared to unfractionated HS (Fig. 7a). While the fractions of < 3 kDa, 3–10 kDa, 10–30 kDa, and 30–100 kDa in FBS could increase PL-MSC growth when compared to the negative control, the proliferation of PL-MSC induced by these fractions was still lower than that induced by unfractionated FBS (Fig. 7a).

Similar to PL-MSCs, the > 100 kDa fraction of FBS could induce a significantly higher number of UC-MSCs compared to unfractionated FBS (Fig. 7b). Although the fractions of < 3 kDa, 3–10 kDa, 10–30 kDa, and 30–100 kDa in FBS could induce UC-MSC growth compared to the negative control, the proliferation of UC-MSC induced by these fractions was still lower than that induced by unfractionated FBS (Fig. 7b).

Taken together, the results suggested that the > 100 kDa fraction of FBS had the highest capacity for inducing MSC proliferation and thus might contain proliferation enhancing factors; therefore, the > 100 kDa fraction of FBS was selected for further analysis.

#### The effects of Concanavalin A fractionated serum on MSC proliferation

The results from the initial serum fractionation suggested that the > 100 kDa fraction of both FBS and HS had the highest effect on MSC growth; therefore, the > 100 kDa fractions of both sera were further fractionated using Concanavalin A (Con-A) lectin affinity chromatography. The effects of Con-A binding proteins and non-Con-A binding proteins on MSC proliferation were then investigated. The > 100 kDa fraction served as a control. At day 3, the number of PL-MSCs cultured in both Con-A binding proteins and non-Con-A binding fractions from FBS were similar to that of PL-MSCs cultured in the > 100 kDa fraction. From day 5 onward, the number of PL-MSCs cultured in Con-A binding proteins was significantly increased compared to non-Con-A binding proteins and the > 100 kDa fraction. At day 10, Con-A binding proteins from FBS induced proliferation of PL-MSCs compared to the > 100 kDa fraction and non-Con-A binding proteins; however, the proliferation of PL-MSCs induced by this fraction was still lower than that induced by 10% FBS (Fig. 8a). Similar to PL-MSCs, Con-A binding proteins from FBS induced higher numbers of UC-MSCs compared to the > 100 kDa fraction and non-Con-A binding proteins. However, the number of UC-MSCs induced by Con-A binding fraction was still lower than that induced by 10% FBS (Fig. 8b).

**Fig. 8:** The effect of Con-A fractionated FBS (**a**, **b**) and HS (**c**, **d**) on MSC proliferation. MSCs were cultured in DMEM+ 5% serum supplemented with either Con-A binding proteins or non-Con-A binding proteins. MSCs cultured in DMEM+ 5% serum supplemented by the > 100 kDa fraction serum served as a control. The cells were harvested at days 3, 5, 7, and 10 to determine the cell numbers. Data are presented as mean ± SEM from three independent experiments. *p < 0.05 compared to control

In contrast to FBS, non-Con-A binding proteins from HS induced higher numbers of PL-MSCs compared to the > 100 kDa fraction and Con-A binding proteins; however, the number of PL-MSCs induced by this fraction was still lower than that induced by 10% HS (Fig. 8c). Furthermore, non-Con-A binding proteins from HS induced higher proliferation of UC-MSC compared to the > 100 kDa fraction and Con-A binding proteins; however, the number of UC-MSCs induced by this fraction was still lower than that induced by 10% HS (Fig. 8d).

#### The effects of Wheat Germ Agglutinin fractionated serum on MSC proliferation

Besides Con-A fractionation, the > 100 kDa fractions of HS were also fractionated using Wheat Germ Agglutinin (WGA) lectin affinity chromatography. The effects of WGA binding proteins and non-WGA binding proteins on MSC growth were then investigated. The > 100 kDa fraction served as a control. At day 3, the number of PL-MSCs cultured in both WGA binding proteins and non-WGA binding proteins was not different to that of PL-MSCs cultured in the > 100 kDa fraction. From day 5 onward, the number of PL-MSCs cultured in WGA binding proteins was significantly increased compared to non-WGA binding proteins. At day 10, WGA binding proteins from HS induced higher number of PL-MSCs compared to non-WGA binding proteins. Interestingly, WGA binding proteins from HS increased PL-MSCs numbers to a similar degree of the > 100 kDa fraction; however, the number of PL-MSCs induced by this fraction was still lower than that induced by 10% HS (Fig. 9a). Together with PL-MSCs, WGA binding proteins from HS increased UC-MSC proliferation to a similar degree of the > 100 kDa fraction. Interestingly, WGA binding proteins from HS induced higher numbers of UC-MSCs compared to non-WGA binding proteins; however, the proliferation of UC-MSCs induced by this fraction was still lower than that induced by 10% HS (Fig. 9b).

**Fig. 9:** The effect of WGA fractionated HS on PL-MSC (**a**) and UC-MSC (**b**) proliferation. MSCs were cultured in DMEM+ 5% serum supplemented with either WGA binding proteins or non-WGA binding proteins. The > 100 kDa HS served as a control. The cells were harvested at days 3, 5, 7, and 10 to determine the cell numbers. Data are presented as mean ± SEM from three independent experiments. *p < 0.05 compared to control

Taken together, the proliferation enhancing factors in FBS might be the Con-A binding proteins in the > 100 kDa fraction. In contrast to FBS, the proliferative enhancing factors in HS might be the non-Con-A binding proteins and WGA binding proteins in the > 100 kDa fraction.

## Discussion

Numerous evidences suggested that MSCs may serve as a promising tool for therapeutic application in various incurable diseases. Therefore, in vitro expansion of MSCs seems to be inevitable due to the requirement of sufficient numbers of MSCs for cell therapy, particularly in relation to clinical applications. For example, a patient with graft versus host disease (GvHD) needs more than 1 × 10^6^ MSCs/kg for infusion. In this regard, the selection of the most appropriate reagents to promote cell proliferation is a critical factor. Currently, the expansion of MSCs has been performed under different culture conditions, most of which were based on the addition of FBS as a supplement. [27]. However, some risks associated with the use of FBS in clinical settings have been raised in terms of potential disease transmission and immunologic reactions. A previous study revealed that anti-FBS antibodies have been detected in most patients infused with MSCs cultured in the presence of FBS [18]. Because of these safety issues for clinical use, the increasing number of clinical protocols emphasizes the need for serum sources or supplements other than FBS. Recently, defined serum-free and xeno-free culture systems have been developed to avoid animal-derived reagents [20, 28]. Nevertheless, certain factors of serum-and xeno-free culture systems have not been fully elucidated [29]. A recent study reported that the existing serum-free medium does not adequately support the proliferation of MSCs in the absence of exogenous growth factors [30]. Therefore, the isolation and initial expansion of MSCs still needs to be carried out using serum-containing medium [20, 28]. In addition, the differentiation of MSCs also requires a serum-containing medium [29]. Therefore, the use of serum for the expansion of MSCs still remains a crucial matter. A previous study showed that HS can be substituted for FBS for MSC expansion [18]. HS-supplemented media significantly increased the number of MSCs without affecting their immunogenicity and oncogenic potential. To the best of our knowledge, this is the first study that directly compared HS and FBS for the isolation and initial expansion of PL-MSCs and UC-MSCs. Remarkably, PLMSCs and UC-MSCs cultured in HS-supplemented medium have similar biological characteristics to PLMSCs and UC-MSCs cultured in FBS-supplemented medium in terms of morphology, immunophenotype, and differentiation capacity [31]. Correspondingly, a previous study, mostly on BM-MSCs, reported similar phenotypic and functional characteristics of MSCs expanded in HS- and in FBS-supplemented media [32].

Flow cytometry analysis indicated that PL-MSCs and UC-MSCs cultured in HS-supplemented medium expressed high levels of MSC markers including the matrix receptor, CD105, and the integrin markers, CD73 and CD90, similar to PL-MSCs and UC-MSCs cultured in FBS-supplemented medium. In addition, PL-MSCs and UC-MSCs cultured in HS-supplemented medium did not express hematopoietic markers including CD34 and CD45 similar to PL-MSCs and UC-MSCs cultured in FBS-supplemented medium [33]. The results suggested that the immunophenotypic characteristics of MSCs cultured in HS-supplemented medium are not different from those of MSCs cultured in FBS-supplemented medium.

Interestingly, PL-MSCs and UC-MSCs cultured in HS-supplemented medium have significantly higher expansion capacities than PL-MSCs and UC-MSCs cultured in FBS-supplemented medium. These results are consistent with a previous study which reported that human BM-MSCs cultured in HS-supplemented medium have a higher proliferative capacity than those cultured in FBS-supplemented medium. BM-MSCs cultured in HS-supplemented medium have shorter population doubling times than those of the cells cultured in FBS-supplemented medium (41–54 h vs. 76–89 h) [27]. It might be possible that HS contains bioactive molecules such as growth factors that are more appropriate to activate human MSCs expansion and function than molecules from FBS [34]. A previous study reported that umbilical cord blood serum is a rich source of growth factors that support proliferation of stem cells. BM-MSCs cultured in umbilical cord blood serum supplemented medium exhibited a 32-fold increase in cell number whereas MSCs cultured in FBS exhibited only 10-fold increase in cell number after seeding for 5 days [35]. In this previous study, hemocomponent supplemented medium could enhance the expansion of MSCs more than 2-fold in the same time when compared to FBS-supplemented medium. The results obtained suggest that HS-supplemented medium has a significantly greater capacity to maintain and expand MSCs than FBS-supplemented medium. Therefore, HS-supplemented medium can be used for MSC expansion with less concern about xenogeneic transmission. Moreover, HS can be used as an autologous serum for MSC expansion in therapeutic applications [36].

In terms of immunosuppressive function, PL-MSCs and UC-MSCs cultured in HS-supplemented medium have a similar degree of immunosuppressive capacity compared to MSCs cultured in FBS-supplemented medium. Generally, PL-MSCs and UC-MSCs cultured in HS-supplemented medium showed a similar immunosuppressive gene expression profile to PL-MSCs and UC-MSCs cultured in FBS-supplemented medium. However, some differences were also observed for the expression of *iNOS*. PL-MSCs and UC-MSCs cultured in HS-supplemented medium highly expressed *IDO* similar to MSCs cultured in FBS-supplemented medium especially when treated with IFN-γ. A previous study revealed that MSCs can suppress T cells proliferation by nonspecific anti-proliferative soluble factors such as IDO, prostaglandin E_2_ (PGE_2_), nitric oxide (NO), transforming growth factor-β (TGF-β), and interleukin-1β (IL-1β) [37]. Among these, IDO and COX2, a key enzyme in the biosynthesis of PGE_2_ [38], are consistently reported as the critical mediators of the immunosuppressive effect of human MSCs [39, 40]. In the mouse, iNOS, a key enzyme in the biosynthesis of NO [41] is reported as the main mediator of the immunosuppressive effect of MSCs [41]. In this study, PL-MSCs and UC-MSCs cultured in FBS-supplemented medium expressed higher iNOS level than MSCs cultured in HS-supplemented medium. In contrast, after treatment with IFN-γ, PL-MSCs and UC-MSCs cultured in HS-supplemented medium had a higher level of *iNOS* expression than MSCs cultured in FBS-supplemented medium. In rats, Burke *et al.* (2014) reported that IFN-γ was not a key factor for inducing *iNOS* expression, but IFN-γ could improve the efficiency of IL-1β to enhance the expression of *iNOS* [42]. It might be possible that IFN-γ is not a key stimulator for *iNOS* expression in human MSCs. Recent studies have shown that the inhibition of T cell proliferation by BMMSCs appeared to be mediated by both cell-cell interaction [43] and the release of soluble factors such as IFN-γ [40, 44]. The result from this study supports a crucial role of IFN-γ in the immunosuppressive capacity of MSCs [40]. The addition of IFN-γ could significantly activate *IDO* expression in PL-MSCs and UC-MSCs. Furthermore, the protein expression exhibited a similar profile as gene expression. Interestingly, MSCs cultured in either HS- or FBS-supplemented medium and stimulated with IFN-γ showed significantly higher IDO expression than that of MSCs stimulated with activated T cells. These results suggest that the expression of IDO from these MSCs might be induced by IFN-γ released from activated T cells [45].

Human serum contains a wide array of proteins and 10% of these serum proteins are glycosylated proteins. After removal of high abundance proteins such as albumin, at least 50% of the remaining proteins are glycoproteins [46]. To identify the proliferation enhancing factors in HS compared to FBS, the serum was fractionated based on molecular weight into five distinct fractions, < 3 kDa, 3–10 kDa, 10–30 kDa, 30–100 kDa, and > 100 kDa. The results showed that the > 100 kDa fraction of both HS and FBS dramatically enhanced the proliferation of PL-MSCs and UC-MSCs when compared to the other fractions.

After this initial fractionation, both HS and FBS were further fractionated using Concanavalin A (Con-A) and Wheat Germ Agglutinin (WGA) lectin affinity chromatography. The results revealed that the candidate proliferation enhancing factors in HS and FBS are different. In FBS, the Con-A binding fraction significantly enhanced the proliferation of PL-MSCs and UC-MSCs. In contrast, in HS only the Con-A flow-through and WGA binding fractions significantly enhanced the proliferation of PL-MSCs and UC-MSCs. Thus, the proliferation enhancing factors in HS are either *N*-acetyl glucosaminylated or sialated groups [47]. Sparbier *et al*. [48] showed that glycosylated or mannosylated proteins could enhance the proliferation of MSCs. Fractionation of HS by lectin affinity chromatography identified 18 glycoproteins from human serum binding to Con-A and 13 glycoproteins binding WGA. Among these, three proteins including alpha-2-macroglobulin, Ceruloplasmin, and a Histidine-rich glycoprotein bind to both Con-A and WGA [30, 48]. Further studies are required to identify the specific proliferation enhancing factors in both HS and FBS, as well as their exact roles.

## Conclusion

This is the first study that compares HS- and FBS-supplemented media for the isolation and expansion of PL-MSCs and UC-MSCs. Our results demonstrate that MSCs cultured in HS-supplemented medium maintain the MSC characteristics and immunosuppressive function similar to MSCs cultured in FBS-supplemented medium. Importantly, MSCs cultured in HS-supplemented medium proliferated better than MSCs cultured in FBS-supplemented medium under the same conditions. Interestingly, the proliferation enhancing factors in HS bind to WGA and do not bind to Con-A, while the reverse is observed in FBS.

Taken together, HS-supplemented medium appears more suitable for MSC isolation and expansion than FBS-supplemented medium. Our initial characterization of the proliferation enhancing factors in HS should lead to a better understanding of the defined factors responsible for this effect. Furthermore, the identification of these factors should help in developing better procedures and culture media for the in vitro expansion of MSCs for clinical applications in the future.

## Abbreviations

1-MT: 1-Methyl-L tryptophan
CD: Cluster of differentiation
cDNA: Complementary deoxyribonucleic acid
CO_2_: Carbon dioxide
COX-2: Cyclooxygenase-2
DMEM: Dulbecco’s modified Eagle’s medium
FBS: Fetal bovine serum
FITC: Fluorescein isothiocyanate
GAPDH: Glyceraldehyde-3-phosphate dehydrogenase
GvHD: Graft versus host disease
HLA: Human leukocyte antigen
HS: Human serum
HSCT: Hematopoietic stem cell transplantation
IDO: Indoleamine 2,3-dioxygenase
IFN-γ: Interferon gamma
IgG: Immunoglobulin G
IL-1β: Interleukin-1 β
iNOS: Inducible nitric oxide synthase
MNCs: Mononuclear cells
MSCs: Mesenchymal stromal cells
NO: Nitric oxide
PB: Peripheral blood
PB-MNCs: Peripheral blood mononuclear cells
PBS: Phosphate-buffered saline
PE: Phycoerythrin
PGE2: Prostaglandin E2
PHA: Phytohemagglutinin
PL: Placenta
PL-MSCs: Placenta-derived mesenchymal stromal cells
qRT-PCR: Quantitative reverse transcriptase polymerase chain reaction
SEM: Standard error of means
TGF-β: Transforming growth factor beta
UC: Umbilical cord
UC-MSCs: Umbilical cord-derived mesenchymal stromal cells
